# Identification of Potential Poly (ADP-Ribose) Polymerase-1 Inhibitors Derived from *Rauwolfia serpentina*: Possible Implication in Cancer Therapy

**DOI:** 10.1155/2022/3787162

**Published:** 2022-03-23

**Authors:** Adel M. Abuzenadah, Fatin Al-Sayes, Syed Sahajada Mahafujul Alam, Mehboob Hoque, Sajjad Karim, Ibtessam M. R. Hussain, Shams Tabrez

**Affiliations:** ^1^Department of Medical Laboratory Science, Faculty of Applied Medical Sciences, King Abdulaziz University, Jeddah, Saudi Arabia; ^2^King Fahd Medical Research Center, King Abdulaziz University, Jeddah, Saudi Arabia; ^3^Center of Excellence in Genomic Medicine Research (CEGMR), King Abdulaziz University, Jeddah, Saudi Arabia; ^4^Applied Bio-Chemistry Lab, Department of Biological Sciences, Aliah University, Kolkata, India

## Abstract

Poly (ADP-ribose) polymerase-1 (PARP-1) has been recognized as a prospective target for the development of novel cancer therapeutics. Several PARP-1 inhibitors are currently being considered for anticancer drug development and clinical investigation. Lately, natural compounds seem to be excellent alternative drug candidates for cancer treatment. *Rauwolfia serpentina* is a medicinal plant traditionally used in Indian subcontinents to treat various diseases. This study has been designed to identify the bioactive compounds derived from *R. serpentina* for possible binding and inhibition of PARP-1 using the molecular docking approach. Thirteen compounds were found to interact with the target with a binding affinity greater than the value of −9.0 kcal/mol. After screening the physicochemical properties, only 5 ligands (ajmalicine, yohimbine, isorauhimbine, rauwolscine, and 1,2-dihydrovomilenine) were found to obey all the parameters of Lipinski's rule of five, showed maximum drug-likeness, and possess no significant toxicity. These ligands displayed strong interactions with target PARP-1 via several hydrogen bonds and hydrophobic interactions. Therefore, these identified compounds derived from *R. serpentina* can be considered for drug development against cancer-targeting PARP-1.

## 1. Introduction

Poly (ADP-ribose) polymerase 1 (PARP-1) is a nuclear enzyme that catalyzes the polymerization of ADP-ribose units obtained from NAD^+^. This helps attach the linear or branched poly (ADP-ribose) (PAR) polymers to itself or other target proteins [1]. This poly (ADP)ribosylation (PARylation) activity of PARP-1 helps perform various functions such as DNA repair of both single-strand and double-strand breaks, stabilization of DNA replication forks, and modification of chromatin structure [1]. PARP-1 has a well-preserved structural and functional organization, comprising three key domains: (1) a double zinc-finger DNA binding domain (DBD) at the amino terminus, required to bind to single-strand and double-strand DNA breaks; (2) a central automodification domain, containing glutamate and lysine residues in the core that act as ADP-ribose moiety acceptors, allowing the enzyme to poly (ADP-ribosyl)ate itself; this region also contains a BRCA1 carboxy-terminal (BRCT) repeat motif and (3) an NAD^+^ binding, catalytic domain with a carboxyl terminus [2, 3].

Accumulating data suggest the overexpression of PARP-1 in several cancer types, including malignant melanomas, neuroblastoma, colorectal cancer, breast cancer, HPV-positive oropharyngeal carcinoma, gastric cancer, testicular and germ cell tumors, malignant lymphoma, and Ewing's sarcoma [4–11]. Therefore, PARP-1 is considered an important target for anticancer therapeutic development. Several drugs have been approved, and many potential drugs targeting PARP-1 are currently under investigation, including some combination therapy [12].

Natural sources are considered a safe pool of potential cancer therapeutics as they pose little risk of harm, unlike the conventional chemotherapeutic agents [13–17]. *Rauwolfia serpentina* is a widely used medicinal plant native to the Indian subcontinent shown to be effective in the treatment of various diseases, including hypertension, intestinal disorders, eye diseases, cuts, wounds, splenic diseases, uterine contraction, headache, and skin disease [18, 19]. It is the bioactive compounds that contribute to the therapeutic activity of the medicinal herbs. The individual compounds display superior medicinal properties, and therefore, identification of the drug-like compounds is essential for novel therapeutic development. This study explores the bioactive compounds derived from *R. serpentina* for their appropriateness as possible PARP-1 inhibitors using the molecular docking technique.

## 2. Materials and Methods

### 2.1. Preparation of Ligand

The 3D structures of the bioactive compounds derived from *R. serpentina* were retrieved from the IMPPAT database (https://cb.imsc.res.in/imppat/home) in SDF format [20]. All atomic coordinates were changed to .pdbqt setup using Open Babel GUI, an open-source chemical toolbox for the interconversion of chemical structures [21].

### 2.2. Preparation of Target Protein

The 3D structure of the target protein PARP-1 was retrieved from the Protein Data Bank (https://www.rcsb.org/) (PDB ID:6I8M). The protein was then prepared for molecular docking studies, the heteroatoms (water and ions) removed, polar hydrogen added, and Kollman charges were assigned. To demarcate the active sites, grid boxes of appropriate sizes were put around the bound cocrystal ligand.

### 2.3. Molecular Docking

Using the AutoDock 4.2 program, the bioactive compounds of *R. serpentina* were docked against PARP-1 molecular target following the previously published procedure [22, 23]. For this, the Lamarckian Genetic Algorithm was used, with the following parameters: a beginning population of 150 randomly inserted individuals, a maximum number of 2,500,000 energy assessments, a mutation rate of 0.02, and a crossover rate of 0.8. A total of 50 independent dockings were performed for each ligand. The grid box's center points were X:6.610, Y:23.444, and Z:20.261, and the dimensions were X:70, Y:70, and Z:70. The grid point spacing was 0.375 Å. The conformations with the lowest binding free energy (ΔG) and the lowest inhibition constant (Ki) were considered the most appropriate. The molecular interactions of the selected ligands with the receptor were evaluated using BIOVIA Discovery Studio [24].

### 2.4. Physicochemical Properties of the Ligands

To assess the tenacity of the compounds showing strong binding affinities for the target protein, the physicochemical properties such as toxicity and drug-likeness were analyzed using the DataWarrior program, version 5.5.0 [25]. The drug-likeness of the selected compounds was examined based on breaches of Lipinski's rule of five [26]. Ligands with zero violations are considered the best drug candidates.

## 3. Results and Discussion

The traditionally used medicinal herb *R. serpentina* has been reported to possess anticancer properties [27]. Previously, the potential antiangiogenic bioactive compounds of *R. serpentina* were identified by targeting VEGFR-2 using the molecular docking approach [22]. Molecular docking is a reliable technique used for *in silico* prediction of potential drug-like compounds for various diseases by targeting certain specific proteins [16, 28–32]. In this study, to identify the potential drug candidates that can effectively bind and inhibit the PARP-1, all the bioactive compounds derived from *R. serpentina* were subjected to molecular docking against the target protein using AutoDock 4.2. Before performing the molecular docking studies, we performed a redocking experiment to test the appropriateness of the docking technique and algorithm. In all cases, the root mean square deviation (RMSD) between docked and native cocrystal locations was less than 2Å which validated our docking parameters [33]. A number of compounds showed strong binding affinities for the target protein. To identify the best drug candidates derived from *R. serpentina*, the binding energy (ΔG) of −9.0 kcal/mol was set as a threshold, and the conformations only with stronger binding energy were selected for further analysis. Out of total 25 compounds of *R. serpentina*, 13 compounds were found to show binding energy below the set threshold. The molecular docking results of the selected ligands against the target protein showing their binding energy (ΔG), minimum inhibition constant (Ki), and interacting amino acid residues are shown in Table 1. Moreover, the exclusive results showing the values of ΔG and Ki for all the *R. serpentina* compounds are presented in Supplementary Table 1. The selected compounds that showed best binding with PARP-1 were found to be serpentinine (ΔG = −14.36 kcal/mol), rescinnamine (ΔG = −10.78 kcal/mol), rescinnamidine (ΔG = −10.71 kcal/mol), phytosterols (ΔG = −10.67 kcal mol), ajmalimine (ΔG = −10.6 kcal/mol), deserpidine (ΔG = −10.17 kcal/mol), ajmalicine (ΔG = −9.75 kcal/mol), reserpine (ΔG = −9.73 kcal/mol), renoxidine (ΔG = −9.66 kcal/mol), yohimbine (ΔG = −9.45 kcal/mol), isorauhimbine (ΔG = −9.39 kcal/mol), rauwolscine (ΔG = −9.1 kcal/mol), and 1,2-dihydrovomilenine (ΔG = −9.08 kcal/mol).

The physicochemical properties of these selected ligands were studied by using DataWarrior program, version 5.5.0, to determine the toxicity and drug-likeness of the compounds [25]. Lipinski's rule of five is conveniently used as the thumb rule to evaluate the “drugability” of new molecular entities based on their pharmacological activities and suggest the possible oral administration of the drug candidates in humans [34]. According to this rule, the absorption or the uptake of a drug candidate is unlikely when it possesses more than 5 H-bond donors, 10 H-bond acceptors, and molecular weight larger than 500 Da and the estimated Log *P* (cLog *P*) is greater than 5 [35]. The results showing various physicochemical parameters of the selected 13 compounds are presented in Table 2. Out of these, only five compounds were found to obey Lipinski's rule of five. The compounds ajmalicine, yohimbine, isorauhimbine, rauwolscine, and 1,2-dihydrovomilenine followed Lipinski's rule of five in all the parameters. However, despite showing good binding affinities and low Ki values (Table 1), the compounds serpentinine, rescinnamine, rescinnamidine, ajmalimine, phytosterols, deserpidine, reserpine, and renoxidine violated Lipinski's rule of five (Table 2).

Serpentinine, the best docked compound of the present study, obeyed Lipinski's rule of five in all the parameters except that it has a molecular weight of 685.842, which is higher than the recommended limit of 500. Moreover, it is nonmutagenic, nontumorigenic, nonirritant, and safe to reproductive health and shows positive drug-likeness. Other physicochemical parameters including topological surface area (TPSA) and the number of rotatable bonds (RB) were found to be within acceptable limits (TPSA ≤ 140Å^2^ and RB ≤ 10) [36]. Similarly, among the selected compounds, rescinnamine, rescinnamidine, phytosterols, deserpidine, reserpine, and renoxidine fail to comply with the guidelines of Lipinski's rule of five in at least one of the set criteria. The compounds rescinnamine, rescinnamidine, reserpine, and renoxidine violated Lipinski's rule of five in multiple parameters such as all of them possess molecular weights greater than 500, more than 10 H-bond acceptors, and rotatable bonds and show a high adverse effect on reproductive health. Ajmalimine and deserpidine have a molecular weight greater than 500, and thus, they violate the rule. The phytosterols have a cLog *P* value of 7.8552, which is higher than the recommended limit indicating poor absorption.

The selected ligands identified against PARP-1 were closely analyzed for their molecular interactions with the target protein (Table 1). The interactions of the best druggable ligands identified based on their physicochemical analysis are discussed here in detail. However, the interactions of those ligands that violated Lipinski's rule of five are also discussed in the subsequent section considering their implication in drug designing. Among the lead drug candidates, ajmalicine was shown to be the best docked to PARP-1 with a ΔG of −9.75 kcal/mol and Ki of 71.69 nM, introducing two hydrogen bonds through His862 and Gly863 and other important and hydrophobic interactions via residues Gln763, Ser864, Ile872, Leu877, Arg878, Ile879, Tyr896, Phe897, Ala880, Gly894, Ile895, Ala898, Lys903, Ser904, and Tyr907 (Figure 1). The strong binding affinity and low Ki value suggest the possible therapeutic implication of ajmalicine in cancer treatment by targeting PARP-1. Previous studies also reported certain therapeutic properties of the alkaloid ajmalicine. It is known to possess antihypertensive activity [37]. Recent studies also demonstrated the therapeutic potential of ajmalicine in Alzheimer's disease (AD) by interacting and inhibiting multiple targets [38].

Another ligand, yohimbine was found to be the best docked to PARP-1 with a ΔG of −9.45 kcal/mol and a Ki of 117.83 nM, introducing four hydrogen bonds through Asp770, His862, Gly863, and Ser864 and additional significant and hydrophobic contacts via residues Gln763, Asp766, Asn767, Asn868, Ile872, Leu877, Arg878, Ile895, Tyr896, Phe897, Ala898, Ser904, and Tyr907 (Figure 2). Yohimbine is an antagonist of *α*2-adrenergic receptor, which is reported to exhibit inhibitory activity against breast cancer and pancreatic cancer cell proliferation [39–41]. In our previous study, we observed a strong binding affinity of yohimbine against VEGFR-2 implicating its potential role in the inhibition of angiogenesis [22].

The ligand isorauhimbine was found to interact with target PARP-1, with a ΔG of −9.39 kcal/mol and a Ki of 130.34 nM, introducing three hydrogen bonds through Asn767, Arg878, and Ala880, as well as other significant and hydrophobic contacts via residues Ile872, Gln763, Asp766, Asp770, His862, Gly863, Ser864, Arg865, Asn868, Leu877, Ile879, Gly894, Ile895, Tyr907, and His909 (Figure 3). These findings suggest the potential of this indole alkaloid in cancer drug development.

Rauwolscine was found to bind at the best pose to PARP-1 with a ΔG of −9.1 kcal/mol and a Ki of 212.64 nM, involving two hydrogen bonds via Gly888 and Met890, as well as additional significant and hydrophobic contacts through residues Trp861, His862, Gly863, Tyr889, Phe891, Tyr896, Ser804, Phe897, Ala898, Lys903, Tyr907, and Glu988 (Figure 4). Like yohimbine, rauwolscine is also a known antagonist of *α*2-adrenergic receptor with potential anticancer and antiangiogenic activity [22].

Another ligand 1,2-dihydrovomilenine was found to be the best docked to PARP-1, with a ΔG of −9.08 kcal/mol and a Ki of 219.89 nM, introducing a single hydrogen bond via residue Gln763, as well as other hydrophobic contacts via residues Trp861, His862, Gly863, Ser864, Asn868, Tyr896, Phe897, Ala898, Lys903, Ser904, Tyr907, and Glu988 (Figure 5). These results support the possible anticancer potential of 1,2-dihydrovomilenine by targeting PARP-1. Similarly, a strong binding affinity of this compound with VEGFR-2 has recently been observed, indicating possible antiangiogenic activity [22].

Moreover, the interactions of ligands that disobeyed Lipinski's rule of five but showed strong affinity towards PARP-1 were also studied. This information would help in designing novel molecules to target PARP-1 based on these ligands. The ligand serpentinine was found to interact with target PARP-1, with the highest affinity (ΔG) of −14.36 kcal/mol and the lowest Ki of 29.59 pM, indicating its strong inhibition efficacy. Serpentinine interacts with PARP-1 by forming five hydrogen bonds through His862, Gly863, Ser864, Asn868, and Gly894, as well as other significant and hydrophobic contacts via residues Gln763, Asp766, Asn767, Trp861, His862, Ile872, Leu877, Arg878, Ala880, Gly888, Tyr889, Met890, Gly894, Ile895, Tyr896, Phe897, Ala898, Glu988, Lys903, Ser904, and Tyr907 (Supplementary Figure S1). The ligand rescinnamine was shown to be the best docked to PARP-1 with a ΔG of −10.78 kcal/mol and Ki of 12.49 nM, introducing three hydrogen bonds through His862, Gly863, and Arg878 and other important and hydrophobic interactions via residues Gln759, Ala760, Val762, Gln763, Asp766, Ser864, Ile872, Leu877, Ile879, Ala880, Gly888, Tyr889, Gly894, Ile895, Tyr896, Phe897, Ala898, Tyr907, Lys908, and Glu988 (Supplementary Figure S2). The ligand rescinnamidine was found to interact with target PARP-1, with a ΔG of −10.71 kcal/mol and a Ki of 14.03 nM, introducing two hydrogen bonds through single amino acid residue Ala880, as well as other significant and hydrophobic contacts via residues Gln759, Gln763, Trp861, His862, Gly863, Arg878, Ile879, Gly888, Tyr889, Lys893, Gly894, Tyr896, Phe897, Ala898, Met890, Ser904, Tyr907, Lys908, and Glu988 (Supplementary Figure S3). Phytosterols were found to interact with target PARP-1, with a ΔG of −10.67 kcal/mol and a Ki of 15.17 nM, introducing two hydrogen bonds through Gly876 and Arg878, as well as other significant and hydrophobic contacts via residues Gln763, Trp861, His862, Gly863, Ser864, Asn868, Ile872, Leu877, Ile895, Tyr896, Phe897, Ala898, Lys903, Ser904, Tyr907, and Glu988 (Supplementary Figure S4). Ajmalimine was shown to be the best docked to PARP-1 with a ΔG of −10.6 kcal/mol and Ki of 17.11 nM, introducing two hydrogen bonds through Gly863 and Gly894 and other important and hydrophobic interactions via residues Asp766, Val762, Gln763, Trp861, His862, Leu877, Arg878, Ile879, Ala880, Tyr889, Lys893, Ile895, Tyr896, Phe897, Ala898, Lys903, Ser904, Tyr907, and Glu988 (Supplementary Figure S5). Deserpidine was found to interact with target PARP-1, with a ΔG of −10.17 kcal/mol and a Ki of 34.86 nM, introducing two hydrogen bonds through Gly888 and Tyr896, as well as other significant and hydrophobic contacts via residues Gln759, Ala760, Val762, Gln763, Asp766, His862, Ile872, Leu877, Arg878, Ile879, Ala880, Tyr889, Gly894, and Ile895 (Supplementary Figure S6). Similarly, reserpine was found to bind at the best pose to the target PARP-1, with a ΔG of −9.73 kcal/mol and a Ki of 73.86 nM, involving two hydrogen bonds via Gln763 and Tyr896, as well as additional significant and hydrophobic contacts through residues Gln759, Val762, Asp770, Ile872, Leu877, Arg878, Ile879, His862, Gly863, Ala880, Gly888, Tyr889, Met890, Gly894, Ile895, and Tyr907 (Supplementary Figure S7). The ligand renoxidine was found to be the best docked to PARP-1, with a ΔG of −9.66 kcal/mol and a Ki of 83.00 nM, introducing three hydrogen bonds via residues Gly888, Met890, and Tyr907, as well as other hydrophobic contacts via residues Gln759, Ala760, Val762, Gln763, Asp766, Trp861, His862, Gly863, Pro885, Thr887, Tyr889, Tyr896, Phe897, Ala898, Ser904, Lys908, and Glu988 (Supplementary Figure S8).

Altogether, in this study, the drug candidates that can potentially bind and inhibit PARP-1 were identified from the bioactive compounds derived from *R. serpentina*. This study also provides insights into the mode of interactions of the ligands with PARP-1. Out of the total 25 constituent compounds, a total of 13 ligands were found to interact with the target with a binding affinity of greater than the threshold value of ΔG = −9.0 kcal/mol. Among these ligands, finally, only five were tested to obey all the parameters of Lipinski's rule of five and show maximum drug-likeness without any display of harmful effects. These are ajmalicine, yohimbine, isorauhimbine, rauwolscine, and 1,2-dihydrovomilenine. They were found to form stable binding with PARP-1 via several hydrogen bonds and hydrophobic interactions. Therefore, all these five compounds can be considered as promising leads for further studies to target PARP-1.

## 4. Conclusion

PARP-1 is an established target for various anticancer therapeutics. The five identified compounds (ajmalicine, yohimbine, isorauhimbine, rauwolscine, and 1,2-dihydrovomilenine) derived from *R. serpentina* with strong binding affinity against PARP-1 display great potential to be considered for anticancer drug development. Moreover, other ligands that showed stable interaction with the studied target and inhibition at a lower concentration can also be considered for drug designing against PARP-1. This study recommends further investigation and validation of the therapeutic efficacy of *R. serpentina* against various forms of cancer in isolation and combination with other drugs so that their potential could be exploited to the maximum.

## Figures and Tables

**Figure 1:** The binding pattern of ajmalicine derived from *R. serpentina* with PARP-1. The (a) 3D and (b) 2D images were generated by using BIOVIA Discovery Studio showing amino acid residues involved in various interactions between PARP-1 and ajmalicine.

**Figure 2:** The binding pattern of yohimbine derived from *R. serpentina* with PARP-1. The (a) 3D and (b) 2D images were generated by using BIOVIA Discovery Studio showing amino acid residues involved in interactions between PARP-1 and yohimbine.

**Figure 3:** The binding pattern of isorauhimbine derived from *R. serpentina* with PARP-1. The (a) 3D and (b) 2D images were generated by using BIOVIA Discovery Studio showing amino acid residues involved in interactions between PARP-1 and isorauhimbine.

**Figure 4:** The binding pattern of rauwolscine derived from *R. serpentina* with PARP-1. The (a) 3D and (b) 2D images were generated by using BIOVIA Discovery Studio showing amino acid residues involved in interactions between PARP-1 and rauwolscine.

**Figure 5:** The binding pattern of 1,2-dihydrovomilenine derived from *R. serpentina* with PARP-1. The (a) 3D and (b) 2D images were generated by using BIOVIA Discovery Studio showing amino acid residues involved in interactions between PARP-1 and 1,2-dihydrovomilenine.

**Table 1:** The binding energy, inhibition constant, and molecular interactions of the selected compounds derived from *R. serpentina* docked against PARP-1.

Sl. no.	Name	Binding energy (kcal/mol)	Ki	Interactive residue	No. of H-bonds and the interactive residues
1	Serpentinine	−14.36	29.59 pM	Gln763, Asp766, Asn767, Trp861, His862, Gly863, Ser864, Asn868, Ile872, Leu877, Arg878, Ala880, Gly888, Tyr889, Met890, Gly894, Ile895, Tyr896, Phe897, Ala898, Glu988, Lys903, Ser904, Tyr907	5; His862, Gly863, Ser864, Asn868, Gly894

2	Rescinnamine	−10.78	12.49 nM	Gln759, Ala760, Val762, Gln763, Asp766, His862, Gly863, Ser864, Ile872, Leu877, Arg878, Ile879, Ala880, Gly888, Tyr889, Gly894, Ile895, Tyr896, Phe897, Ala898, Tyr907, Lys908, Glu988	3; His862, Gly863, Arg878

3	Rescinnamidine	−10.71	14.03 nM	Gln759, Gln763, Trp861, His862, Gly863, Arg878, Ile879, Ala880, Gly888, Tyr889, Lys893, Gly894, Tyr896, Phe897, Ala898, Met890, Ser904, Tyr907, Lys908, Glu988	2; Ala880

4	Phytosterols	−10.67	15.17 nM	Gln763, Trp861, His862, Gly863, Ser864, Asn868, Ile872, Gly876, Leu877, Arg878, Ile895, Tyr896, Phe897, Ala898, Lys903, Ser904, Tyr907, Glu988	2; Gly876, Arg878

5	Ajmalimine	−10.6	17.11 nM	Asp766, Val762, Gln763, Trp861, His862, Gly863, Leu877, Arg878, Ile879, Ala880, Tyr889, Lys893, Gly894, Ile895, Tyr896, Phe897, Ala898, Lys903, Ser904, Tyr907, Glu988	2; Gly863, Gly894

6	Deserpidine	−10.17	34.86 nM	Gln759, Ala760, Val762, Gln763, Asp766, His862, Ile872, Leu877, Arg878, Ile879, Ala880, Gly888, Tyr889, Gly894, Ile895, Tyr896	2; Gly888, Tyr896

7	Ajmalicine	−9.75	71.69 nM	Gln763, His862, Gly863, Ser864, Ile872, Leu877, Arg878, Ile879, Tyr896, Phe897, Ala880, Gly894, Ile895, Ala898, Lys903, Ser904, Tyr907	2; His862, Gly863

8	Reserpine	−9.73	73.86 nM	Gln759, Val762, Gln763, Asp770, Ile872, Leu877, Arg878, Ile879, His862, Gly863, Ala880, Gly888, Tyr889, Met890, Gly894, Ile895, Tyr896, Tyr907	2; Gln763, Tyr896

9	Renoxidine	−9.66	83.00 nM	Gln759, Ala760, Val762, Gln763, Asp766, Trp861, His862, Gly863, Pro885, Thr887, Gly888, Tyr889, Met890, Tyr896, Phe897, Ala898, Ser904, Tyr907, Lys908, Glu988	3; Gly888, Met890, Tyr907

10	Yohimbine	−9.45	117.83 nM	Gln763, Asp766, Asn767, Asp770, His862, Gly863, Ser864, Asn868, Ile872, Leu877, Arg878, Ile895, Tyr896, Phe897, Ala898, Ser904, Tyr907.	4; Asp770, His862, Gly863, Ser864

11	Isorauhimbine	−9.39	130.34 nM	Asn767, Ile872, Gln763, Asp766, Asp770, His862, Gly863, Ser864, Arg865, Asn868, Leu877, Arg878, Ile879, Ala880, Gly894, Ile895, Tyr907, His909	3; Asn767, Arg878, Ala880

12	Rauwolscine	−9.1	212.64 nM	Trp861, His862, Gly863, Tyr889, Phe891, Tyr896, Ser804, Gly888, Met890, Phe897, Ala898, Lys903, Tyr907, Glu988	2; Gly888, Met890

13	1,2-Dihydrovomilenine	−9.08	219.89 nM	Gln763, Trp861, His862, Gly863, Ser864, Asn868, Tyr896, Phe897, Ala898, Lys903, Ser904, Tyr907, Glu988	1; Gln763

**Table 2:** Physicochemical properties of the selected ligands derived from *R. serpentina*.

Sl. no.	Name	Mol weight	cLog *P*	cLog *S*	H-acceptors	H-donors	Polar surface area	Drug-likeness	Mutagenic	Tumorigenic	Reproductive effective	Irritant	Rotatable bonds
1	Serpentinine	685.842	2.4747	−6.147	9	2	100.53	1.3453	None	None	None	None	7
2	Rescinnamine	634.723	3.9046	−4.816	11	1	117.78	0.21574	None	None	High	None	11
3	Rescinnamidine	636.739	4.0279	−4.681	11	1	117.78	-1.0959	None	None	High	None	12
4	Phytosterols	414.715	7.8552	−6.669	1	1	20.23	-4.475	None	None	None	None	6
5	Ajmalimine	520.624	3.5094	−5.118	8	1	80.7	3.4909	None	None	None	Low	7
6	Deserpidine	578.66	3.6454	−4.428	10	1	108.55	2.322	None	None	None	None	9
7	Ajmalicine	352.433	2.2674	−3.141	5	1	54.56	2.6043	None	None	None	None	2
8	Reserpine	608.686	3.5754	−4.446	11	1	117.78	2.322	None	None	High	None	10
9	Renoxidine	624.685	2.602	−2.277	12	1	131.61	-2.8747	None	None	High	None	10
10	Yohimbine	354.448	2.3512	−3.065	5	2	65.56	1.5035	None	None	None	None	2
11	Isorauhimbine	354.448	2.3512	−3.065	5	2	65.56	1.5035	None	None	None	None	2
12	Rauwolscine	354.448	2.3512	−3.065	5	2	65.56	1.5035	None	None	None	None	2
13	1,2-Dihydrovomilenine	352.433	1.8244	−3.654	5	2	61.8	1.1872	None	None	None	None	2

## Data Availability

Data are available on request to the corresponding author.

## Supplementary Materials

Supplementary Materials Supplementary Figure S1: the binding pattern of serpentinine derived from *R. serpentina* with the PARP-1. The 3D and 2D images were generated by using BIOVIA Discovery Studio showing amino acid residues involved in interactions between PARP-1 and serpentinine. Supplementary Figure S2: the binding pattern of rescinnamine derived from *R. serpentina* with the PARP-1. The 3D and 2D images were generated by using BIOVIA Discovery Studio showing amino acid residues involved in interactions between PARP-1 and rescinnamine. Supplementary Figure S3: the binding pattern of rescinnamidine derived from *R. serpentina* with the PARP-1. The 3D and 2D images were generated by using BIOVIA Discovery Studio showing amino acid residues involved in interactions between PARP-1 and rescinnamidine. Supplementary Figure S4: the binding pattern of phytosterols derived from *R. serpentina* with the PARP-1. The 3D and 2D images were generated by using BIOVIA Discovery Studio showing amino acid residues involved in interactions between PARP-1 and phytosterols. Supplementary Figure S5: the binding pattern of ajmalimine derived from *R. serpentina* with the PARP-1. The 3D and 2D images were generated by using BIOVIA Discovery Studio showing amino acid residues involved in interactions between PARP-1 and ajmalimine. Supplementary Figure S6: the binding pattern of deserpidine derived from *R. serpentina* with the PARP-1. The 3D and 2D images were generated by using BIOVIA Discovery Studio showing amino acid residues involved in interactions between PARP-1 and deserpidine. Supplementary Figure S7: the binding pattern of reserpine derived from *R. serpentina* with the PARP-1. The 3D and 2D images were generated by using BIOVIA Discovery Studio showing amino acid residues involved in interactions between PARP-1 and reserpine. Supplementary Figure S8: the binding pattern of renoxidine derived from *R. serpentina* with the PARP-1. The 3D and 2D images were generated by using BIOVIA Discovery Studio showing amino acid residues involved in interactions between PARP-1 and renoxidine.

## References

[1] Ray Chaudhuri A., Nussenzweig A. (2017). The multifaceted roles of PARP1 in DNA repair and chromatin remodelling. *Nature Reviews Molecular Cell Biology*.

[2] Kraus W. L., Lis J. T. (2003). PARP goes transcription. *Cell*.

[3] Rouleau M., Patel A., Hendzel M. J., Kaufmann S. H., Poirier G. G. (2010). PARP inhibition: PARP1 and beyond. *Nature Reviews Cancer*.

[4] Dziaman T., Ludwiczak H., Ciesla J. M. (2014). PARP-1 expression is increased in colon adenoma and carcinoma and correlates with OGG1. *PLoS ONE*.

[5] Liu Q., Ma L., Jones T. (2018). Subjugation of TGF*β* signaling by human papilloma virus in head and neck squamous cell carcinoma shifts DNA repair from homologous recombination to alternative end joining. *Clinical Cancer Research*.

[6] Liu Y., Zhang Y., Zhao Y., Gao D., Xing J., Liu H. (2016). High PARP-1 expression is associated with tumor invasion and poor prognosis in gastric cancer. *Oncology Letters*.

[7] Mego M., Cierna Z., Svetlovska D. (2013). PARP expression in germ cell tumours. *Journal of Clinical Pathology*.

[8] Newman E. A., Lu F., Bashllari D., Wang L., Opipari A. W., Castle V. P. (2015). Alternative NHEJ pathway components are therapeutic targets in high-risk neuroblastoma. *Molecular Cancer Research*.

[9] Newman R., Soldatenkov V., Dritschilo A., Notario V. (2002). Poly(ADP-ribose) polymerase turnover alterations do not contribute to PARP overexpression in ewing’s sarcoma cells. *Oncology Reports*.

[10] Rojo F., García-Parra J., Zazo S. (2012). Nuclear PARP-1 protein overexpression is associated with poor overall survival in early breast cancer. *Annals of Oncology*.

[11] Tomoda T., Kurashige T., Moriki T., Yamamoto H., Fujimoto S., Taniguchi T. (1991). Enhanced expression of poly(ADP-ribose) synthetase gene in malignant lymphoma. *American Journal of Hematology*.

[12] Rose M., Burgess J. T., O’Byrne K., Richard D. J., Bolderson E. (2020). PARP inhibitors: clinical relevance, mechanisms of action and tumor resistance. *Frontiers in Cell and Developmental Biology*.

[13] Alam S. S. M., Uddin F., Khan F. B., Kamal M. A., Hoque M. (2022). Therapeutic and pharmacological potential of tanshinones against lung cancer: a systematic review. *Phytomedicine Plus*.

[14] Damery S., Gratus C., Grieve R. (2011). The use of herbal medicines by people with cancer: a cross-sectional survey. *British Journal of Cancer*.

[15] Uddin F., Hoque M., Tabrez S., Imran Khan M. (2021). Non-flavonoids targeting cancer stem cells: a promising therapeutic avenue for cancer treatment. *Polyphenols-based Nanotherapeutics for Cancer Management*.

[16] Roy A., Anand A., Garg S. (2022). Structure-based in silico investigation of agonists for proteins involved in breast cancer. *Evidence-based Complementary and Alternative Medicine*.

[17] Roy A., Bhatia K. S. (2021). In silico analysis of plumbagin against cyclin-dependent kinases receptor. *Vegetos*.

[18] Dey A., De J. N. (2011). Ethnobotanical aspects of *Rauvolfia serpentina* (L). Benth. ex Kurz. in India, Nepal and Bangladesh. *Journal of Medicinal Plants Research*.

[19] Pathania S., Ramakrishnan S. M., Randhawa V., Bagler G. (2015). SerpentinaDB: a database of plant-derived molecules of *Rauvolfia serpentina*. *BMC Complementary and Alternative Medicine*.

[20] Mohanraj K., Karthikeyan B. S., Vivek-Ananth R. P. (2018). IMPPAT: a curated database of Indian medicinal plants, phytochemistry and therapeutics. *Scientific Reports*.

[21] O’Boyle N. M., Banck M., James C. A., Morley C., Vandermeersch T., Hutchison G. (2011). Open babel: an open chemical toolbox. *Journal of Cheminformatics*.

[22] Abuzenadah A. M., Al-Sayes F., Alam S. S. M. (2022). Elucidating anti-angiogenic potential of *Rauwolfia serpentina*: VEGFR-2 targeting based molecular docking study. *Evidence-Based Complementary and Alternative Medicine*.

[23] Morris G. M., Huey R., Lindstrom W. (2009). AutoDock4 and AutoDockTools4: automated docking with selective receptor flexibility. *Journal of Computational Chemistry*.

[24] BIOVIA (2021). *Dassault Systémes*.

[25] Sander T., Freyss J., von Korff M., Rufener C. (2015). DataWarrior: an open-source program for chemistry aware data visualization and analysis. *Journal of Chemical Information and Modeling*.

[26] Lipinski C. A. (2004). Lead- and drug-like compounds: the rule-of-five revolution. *Drug Discovery Today: Technologies*.

[27] Alshahrani M. Y., Rafi Z., Alabdallah N. M. (2021). A comparative antibacterial, antioxidant, and antineoplastic potential of Rauwolfia serpentina (L.) leaf extract with its biologically synthesized gold nanoparticles (R-AuNPs). *Plants*.

[28] Jabir N. R., Rehman Md. T., Alsolami K. (2021). Concatenation of molecular docking and molecular simulation of BACE-1, *γ*-secretase targeted ligands: in pursuit of Alzheimer’s treatment. *Annals of Medicine*.

[29] Jabir N. R., Shakil S., Tabrez S., Khan M. S., Rehman M. T., Ahmed B. A. (2021). In silico screening of glycogen synthase kinase-3*β* targeted ligands against acetylcholinesterase and its probable relevance to Alzheimer’s disease. *Journal of Biomolecular Structure and Dynamics*.

[30] Jabir N. R., Rehman M. T., Tabrez S. (2021). Identification of butyrylcholinesterase and monoamine oxidase B targeted ligands and their putative application in alzheimer’s treatment: a computational strategy. *Current Pharmaceutical Design*.

[31] Roy A., Menon T. (2021). *Evaluation of Bioactive Compounds from Boswellia Serrata against SARS-CoV-2*.

[32] Garg S., Roy A. (2020). In Silico analysis of selected alkaloids against main protease (Mpro) of SARS-CoV-2. *Chemico-Biological Interactions*.

[33] Januar H., Dewi A., Marraskuranto E., Wikanta T. (2012). In silico study of fucoxanthin as a tumor cytotoxic agent. *Journal of Pharmacy and Bioallied Sciences*.

[34] Lipinski C. A., Lombardo F., Dominy B. W., Feeney P. J. (1997). Experimental and computational approaches to estimate solubility and permeability in drug discovery and development settings. *Advanced Drug Delivery Reviews*.

[35] Benet L. Z., Hosey C. M., Ursu O., Oprea T. I. (2016). BDDCS, the rule of 5 and drugability. *Advanced Drug Delivery Reviews*.

[36] Halim S. A., Waqas M., Khan A., Al-Harrasi A. (2021). In silico prediction of novel inhibitors of SARS-CoV-2 main protease through structure-based virtual screening and molecular dynamic simulation. *Pharmaceuticals*.

[37] Hemmati N., Azizi M., Spina R. (2020). Accumulation of ajmalicine and vinblastine in cell cultures is enhanced by endophytic fungi of *Catharanthus roseus* cv. icy pink. *Industrial Crops and Products*.

[38] Kashyap P., Kalaiselvan V., Kumar R., Kumar S. (2020). Ajmalicine and reserpine: indole alkaloids as multi-target directed ligands towards factors implicated in alzheimer’s disease. *Molecules*.

[39] Luthy I., Bruzzone A., Pinero C. (2009). Adrenoceptors: non conventional target for breast cancer?. *Current Medicinal Chemistry*.

[40] Pérez Piñero C., Bruzzone A., Sarappa M., Castillo L., Lüthy I. (2012). Involvement of *α*2- and *β*2-adrenoceptors on breast cancer cell proliferation and tumour growth regulation: adrenoceptor regulation of mammary tumour growth. *British Journal of Pharmacology*.

[41] Shen S.-G., Zhang D., Hu H.-T., Li J.-H., Wang Z., Ma Q.-Y. (2008). Effects of *α*-adrenoreceptor antagonists on apoptosis and proliferation of pancreatic cancer cells in vitro. *World Journal of Gastroenterology*.

